# Characteristics and Rehabilitation Training Effects of Shoulder Joint Dysfunction in Volleyball Players under the Background of Artificial Intelligence

**DOI:** 10.1155/2022/4512795

**Published:** 2022-06-29

**Authors:** Yunqi Tang, Zhaoyang Chen, Xiangyun Lin

**Affiliations:** ^1^School of Sports Medicine and Rehabilitation, North Sichuan Medical College, Nanchong 637100, Sichuan, China; ^2^Railway Transportation College, Hope College, Southwest Jiaotong University, Chengdu 610400, Sichuan, China

## Abstract

With the development of volleyball technology, the frequent competition, the fierce competition, and the increase of sports load, the requirements for the athletes' own body, intelligence, combat, heart, and skills are getting higher and higher. Volleyball is one of the most popular sports in the world. It attracts people all over the world with its strong team appeal and its own unique charm. This study mainly discusses the characteristics of shoulder joint dysfunction in volleyball players and the effect of rehabilitation training under the background of artificial intelligence. By sorting out the development process of artificial intelligence technology, it can be analyzed that artificial intelligence technology already has a certain knowledge reserve, can make corresponding mechanized feedback, and can make correct judgments based on experience in more complex situations. This study compared volleyball athletes with handicap and barrier-free shoulder joints and observed the characteristics of shoulder pain, stability, and flexibility caused by subacromial impingement syndrome. It also looked at whether subacromial impingement syndrome athletes differ in volleyball spiking sequence and mobilization and recruitment of muscle power during swing spikes compared to athletes with normal shoulder function in the full kinetic chain. According to the volleyball intelligent competition platform, the implementation and application of ideas such as data collection, result feedback, adjustment of training plan, implementation of training plan, and real-time monitoring are regularly monitored. On the one hand, through timely assessment and detection of shoulder function of volleyball players, functional training is carried out for weaknesses to prevent injury; on the other hand, after a mild injury occurs, timely targeted training should be taken to find and correct wrong actions, and strengthen the weak part of muscle strength, so as to reduce the probability of repeated injury and improve sports performance and athletic ability. In the new system, after collecting and sorting, testers can directly upload to the web page in the form of Excel for automatic filling, grasp the test information of athletes in time, generate automatic warning, and save time. The monitoring content determined by this study mainly includes three index systems, including load, training preparation performance, and recovery. According to the self-provided evaluation system of relevant test equipment and the experience of expert coaches, the evaluation standards for each index are formulated. There was a statistically significant difference in the scores between the rehabilitation group and the pre-rehabilitation group during the study (*P* < 0.05). This study attempts to find the characteristics and rules of FMS scores of women's volleyball players of different levels, so as to provide more targeted physical training for volleyball players, promote the all-round development of physical fitness, and avoid the risk of sports injuries. This study provides more effective and comprehensive recommendations for the prevention and recovery of shoulder injuries in volleyball players. This study provides more effective and comprehensive recommendations for the prevention and recovery of shoulder injuries in volleyball players. The results of the study can provide reference for the scientific training and rehabilitation of volleyball players and make suggestions for the treatment and prevention of subacromial impingement syndrome.

## 1. Introduction

In recent years, the theoretical research on risk management has been applied in the field of competitive sports and has achieved fruitful scientific research results and practical results. However, the research on risk management in college physical education teaching is obviously insufficient; in particular, the risk management research in college sports volleyball special teaching is less. From the perspective of the characteristics of volleyball, competitive volleyball, as a comprehensive competitive sport, requires athletes to have comprehensive sports qualities, such as reaction, speed, strength, endurance, flexibility, and coordination.

This study investigates the risk sources and risk factors of sports injuries in sports volleyball special teaching activities and puts forward reasonable suggestions for sports volleyball special teaching activities to deal with sports injury risks. It helps sports volleyball students and physical education teachers to think about sports injuries in volleyball teaching activities from a new perspective. The perfect and rational echelon construction of the women's volleyball team is the cornerstone for the Chinese women's volleyball team to become one of the world's top volleyball teams. Therefore, it is of great practical significance to study the women's volleyball players at three different levels from different angles and at different levels.

In recent years, artificial intelligence has developed rapidly, and its development in the field of sports is even more prominent. In the context of the development of this era, for the hospital outpatient hall space, how to adapt to the general trend of the times faster and better, and continuously provide efficient and high-quality sports services for the society has become an important issue. After the impact injury, the shoulder's balance ability, coordination ability, and sports adaptation ability will decline, so the rehabilitation training needs to include the training to restore the muscle balance around the shoulder joint. At the same time, in order to avoid shoulder injury caused by wrong spiking action to the volleyball players when spiking, in situ spiking and arm swing exercises are also added to the training, while increasing muscle strength can improve the neuromuscular control of the shoulder joint to the spiking action. Muscle is an important part of human body structure and also the power source of human movement. The physical activity is the main body of the human body, and the size of the human muscle strength is directly related to the quality of sports performance.

## 2. Related Work

In volleyball, the basic technical movements such as serving, passing, and padding are mainly performed by the shoulder joint, which is completed through the flexion and extension of the shoulder joint. With the development of volleyball technology, the frequent competition, the fierce competition, and the increase of sports load, the requirements for the athletes' own body, intelligence, combat, heart, and skills are getting higher and higher. Etminaniesfahani et al. introduced a new metaheuristic algorithm. This optimization algorithm was inspired by a very popular tool among technical traders in the stock market called the Fibonacci indicator. Fibonacci indicators are used to predict possible local highs and lows, as well as periods where stock prices will experience a lot of movement. His proposed Fibonacci indicator algorithm has been validated on multiple benchmark functions in up to 100 dimensions and compared with algorithms such as DE extension, PSO extension, ABC, ABC-PS, CS, MCS, and GSA in terms of convergence and finding the global optimum. Finally, the performance of the algorithm is demonstrated through two engineering design problems. The application of the proposed Fibonacci indicator algorithm to a wide range of benchmark functions demonstrates its ability to handle difficult optimization problems [1]. The work by Pomorski and Perche involves fault detection and isolation (FDI) of induction motors. It cannot be supervised with knowledge of analyzing redundant relations alone: the normal operating state of the motor and the speed sensor failure state cannot be distinguished from the behavioral analysis model. He proposes a solution using two inductive learning techniques based on the form of decision trees: C4.5 is a milestone for top-down induction of decision trees, and BUST is a solution to the problem of functional separability of decision trees [2]. Makridakis believes that the impact of the industrial and digital (information) revolution has undoubtedly had a major impact on almost all aspects of society, life, companies, and employment. By studying similar inventions in the industrial, digital, and artificial intelligence revolutions, he claims the latter is the goal, which will bring about widespread changes that will also affect every aspect of society and life. Furthermore, its impact on businesses and employment will be enormous, leading to increased global competition among highly interconnected organizations and businesses based on big data analysis and decision making. People will be able to use the Internet to buy goods and obtain services from anywhere in the world, and take advantage of the unlimited additional benefits brought about by the widespread use of artificial intelligence inventions. Those who use the Internet extensively and are willing to take entrepreneurial risks to turn around will continue to gain a significant competitive advantage [3]. Zhengping et al. proposed a feature fusion method, introduced a metric learning method, and learned a transformation matrix to make the distance between kinship samples smaller and the distance between nonrelative samples larger. The prior knowledge of the similarity of existing data samples is used to learn the best similarity measure to better describe the similarity of relative samples [4]. Zhao et al. believes that 5G cellular networks are considered to be a key enabler and infrastructure provider for the ICT industry, offering a variety of services with different needs. Standardization of 5G cellular networks is accelerating, which also means more candidate technologies will be adopted. Therefore, it is worth digging into the entire candidate technologies and examining the design philosophies behind them. He sought to highlight one of the most fundamental features of the revolutionary technologies of the 5G era, namely, the emergence of initial intelligence in nearly every important aspect of cellular networks, including radio resource management, mobility management, service provisioning management, and more. However, in the face of increasingly complex configuration issues and emerging new service requirements, 5G cellular networks are still not enough if they lack complete AI capabilities. Therefore, he further introduces the fundamental concepts in AI and discusses the relationship between AI and candidate technologies in 5G cellular networks [5]. In the intuitionistic fuzzy environment, Garg proposed a series of average aggregation operators considering the degree of hesitation between membership functions. To this end, some deficiencies of existing aggregation operators are first identified, and then, new operating rules are proposed to overcome these deficiencies. On the basis of these operations, weighted, ordered weighted, and mixed average aggregation operators are proposed using Einstein's algorithm. In addition, some desirable properties, such as idempotency, boundedness, and homogeneity, are also studied. Finally, an operator-based multicriteria decision-making (MCDM) method is proposed and its performance is compared with existing operators [6]. The proprioceptive ability of the shoulder joint and the strength of the muscle strength play a very important role in controlling the stability of the movement. The proprioception and muscle strength are poor, and the shoulder joint is relatively unstable and prone to injury during exercise. Injuries directly affect the training and competition performance of athletes. Techniques and tactics are the premise of winning the game, and physical training is the foundation. How to maintain a good physical state requires training monitoring. Monitoring training has become an important part of an athlete's overall preparation. It is very rare that elite athletes do not do some form of monitoring training, and most elite teams will choose to invest a lot of resources in monitoring systems, making full use of monitoring data to help athletes improve sports performance. Each athlete is an independent individual, and individualized training is established based on this concept. Monitoring training is a two-way regulation process in which the relationship between overtraining and undertraining is reasonably controlled to fully explore the potential of athletes. Due to the rapid development of the Internet, artificial intelligence technology has entered a new era of development. At this stage, artificial intelligence technology has evolved from the stage of knowledge acquisition to the stage of machine learning.

## 3. Characteristics of Shoulder Joint Dysfunction in Volleyball Players under the Background of Artificial Intelligence and Research Methods for Rehabilitation Training

### 3.1. Experimental Grouping

The athletes who performed the experiment were divided into groups: first, the athletes were divided into groups by the SPADI shoulder pain and disability index screening. Players with normal scores (with a score of 0) are in one group, and those with abnormal scores (with a score of not 0) are in other group. The normal score group was randomly divided into two groups: the pre-rehabilitation group and the pre-rehabilitation control group. The pre-rehabilitation group received pre-rehabilitation training and physical training, while the pre-rehabilitation control group received only physical training without intervention. The abnormal score group was randomly divided into two groups: the rehabilitation training group and the rehabilitation control group. The rehabilitation training group carried out active rehabilitation training and physical training, while the rehabilitation control group recovered naturally and only carried out normal physical training. In order to reduce the experimental error, the SPADI shoulder joint pain and function index screening was performed by the same person in the experiment, and the same method was used for muscle release and stretching in the later stage.

### 3.2. Action and Muscle Strength Test

#### 3.2.1. Y-Balance Test

At present, muscle strength test, as a new training testing technology, has been widely used in training and medicine. Because of its high accuracy, safety, and effectiveness, it is known as the “golden method” for evaluating muscle function. To a certain extent, muscle strength testing has opened up a new path for evaluating muscle function, sports rehabilitation, and training.

The main purpose of the upper limb Y-Balance test is to compare and analyze the difference and comprehensive value of the left and right hands in three directions so that it can quickly evaluate the limited dynamic balance, functional symmetry, and injury risk of the upper limbs. When performing the test movement of Y balance, the athlete needs to have neuromuscular control, good flexibility, and sufficient muscle strength. The Y balance test is mainly used to accurately measure the proprioception, joint flexibility, muscle strength, and joint stability required by athletes to complete movements in dynamic balance. This test can be used as one of the predictors of injury risk before injury and can also be used as one of the indicators of whether athletes can resume normal-intensity training after rehabilitation training. In the upper limb Y-Balance test, the difference between the left and right hands in all directions should not be greater than 4 cm, and the respective scores of the left and right hands can reflect the flexibility of the shoulder joint and the stability of the scapula. The smaller the test score, the greater the risk of shoulder injury and vice versa. In order to reduce the experimental error, the Y-Balance test was carried out by the same person in the experiment.

#### 3.2.2. Isokinetic Muscle Strength Test

*American BIODEX isokinetic muscle strength testing system*. The position of the system was set before the test, and the test angular velocity was set to 60°/s and 180°/s, respectively. The test movements include internal rotation, external rotation, adduction, abduction, flexion, and extension of the shoulder joint. Before the action starts, it should adjust the sitting position to ensure that the force is fully exerted. During the test, subjects are required to do their best to complete the entire exercise process. Rest 5 min after each test to avoid fatigue.

According to the total transformation matrix in the positive kinematics solution [7], we have

(1) $$\begin{array}{c} p_{x}=l_{2}\left(c\theta_{1}c\theta_{2}-s\theta_{1}s\theta_{2}\right)+l_{1}c\theta_{1},\\ p_{y}=l_{2}\left(c\theta_{1}c\theta_{2}+c\theta_{2}s\theta_{1}\right)+l_{1}c\theta_{1}. \end{array}$$

At the same time, we square and then add, it can be obtained as follows [8]:

(2) $$\begin{array}{c} p_{x}^{2}+p_{y}^{2}=l_{1}^{2}+l_{2}^{2}+2l_{1}l_{2}. \end{array}$$

*cθ*_2_ can be obtained as follows:

(3) $$\begin{array}{c} c\theta_{2}=\frac{x^{2}+y^{2}-l_{1}^{2}-l_{2}^{2}}{2l_{1}l_{2}},\\ s\theta_{2}=\sqrt{1-{\left(c\theta_{2}\right)}^{2}}. \end{array}$$

It can get *θ*_2_ as follows [9]:

(4) $$\begin{array}{c} \theta_{2}=A\text{tan}2\left(s\theta_{2},c\theta_{2}\right). \end{array}$$

### 3.3. Physical Examination and Scoring Criteria for Subacromial Impingement

1. Neer impact test: the rehabilitation physician stood behind the volleyball player, fixed the scapula on the spiking side with one hand, and kept the shoulder joint on the spiking side in internal rotation with the other hand. Then, let the injured shoulder flex forward until the athlete feels pain or cannot lift up. Pain is in the front or outside of the shoulder, especially when the patient is flexed 90°–140°.
2. Hawkins–Kennedy impact test: let the upper arm on the spiking side of the volleyball player bend forward 90 degrees, elbow flexion 90 degrees, and at the same time, we straighten the forearm without bending. Rehabilitation physicians forced the forearm on the spiking side to internally rotate, and if the athlete felt pain during the examination, it was positive.
3. Infraspinatus test: we have the upper limbs of the volleyball player who flex their elbows 90 degrees together, with the upper limbs in a neutral position and inward to the sides of the body. Rehabilitation physicians force the upper limbs on both sides of the athlete to rotate together, and if the athlete feels weakness or pain, then it is positive.
4. Horizontal adduction test: let the upper limb of the volleyball player on the side of the spiking flex forward 90°, and the rehabilitation doctor will add the upper limb on the side of the spiking to the opposite side. if the athlete experiences shoulder pain, then it is positive.

After finding *θ*_2_, it can be rewritten into the following form [10]:

(5) $$\begin{array}{c} p_{x}=k_{1}c\theta_{1}-k_{2}c\theta_{2},\\ p_{y}=k_{1}s\theta_{1}+k_{2}s\theta_{2}. \end{array}$$

In,

(6) $$\begin{array}{c} k_{1}=l_{1}+l_{2}c\theta_{2},\\ k_{2}=l_{2}s\theta_{2}. \end{array}$$

Then, the calibration problem becomes to find a set of Euclidean transformation *RP*_*i*_ so that the following formula holds [11].

(7) $$\begin{array}{c} \forall_{i,p_{i}}=RP_{i}+t. \end{array}$$

### 3.4. Establishment of an Intelligent Competitive Platform for Volleyball

In terms of data statistical transformation, in the Smartabase system, brands that do not cooperate with cannot achieve digital automatic uploading, and need to export and organize the data in CSV format before uploading. There are also certain problems in the uploading of the training plan by the coaches, and the overall operation is rather cumbersome. Domestic research is underway to address this issue. In the new system, testers can directly upload to the web page in the form of Excel for automatic filling after collecting and sorting. It can save time by grasping the test information of athletes in time and generating automatic warning. The development and application of the system are carried out in line with the principle of convenience and speed.

#### 3.4.1. In Terms of Training Plan

We formulate a daily, weekly, or monthly training plan; import the construction database; create a training plan template that can be used repeatedly; and compare the actual training load and training intensity. On the platform, the training movements selected by the coaches will be displayed with animations. After checking, they can be displayed to the athletes, especially in the movements that need to be completed quickly, so that the athletes can clearly understand the points that need to be paid attention to. At the same time, it can also uploaded the video of the athletes for repeated viewing, found out the problems existing in the training of the athletes, and corrected them in time, so as to achieve visual analysis and timely feedback.

#### 3.4.2. Data Integration Analysis Process

We monitor training and nontraining data collected on a daily basis, and comprehensively analyze all factors that determine success or failure. We identify the parameters with the most predictive value and integrate performance results and personal statistics along with coaching and expertise to create predictive models. It provides daily training regimens that adapt to changing training and environmental conditions by creating interactive tabular content. The system includes the whole solution chart, database module, analysis and classification module, prediction model module, and end-user solution module. The pass classification of the system is shown in Figure 1.

### 3.5. Rehabilitation and Pre-Rehabilitation Training

Functional training methods are mainly used to improve joint stability, neuromuscular regulation, muscle strength, and muscle endurance of injured people; in the field of competitive sports rehabilitation, it is mainly to restore athletes to normal state, relieve pain, and prevent the occurrence of injuries. Volleyball players were divided into 4 groups according to their shoulder pain and disability index. Rehabilitation training group, rehabilitation training control group, pre-rehabilitation group, and pre-rehabilitation control group were trained for 4 weeks, and all four groups were given normal physical training. The rehabilitation training group did about 60 minutes of rehabilitation training every Monday, Wednesday, and Friday, and the pre-rehabilitation group did about 60 minutes of intervention training every Monday, Wednesday, and Friday. Finally, the differences in the sports performance of the three were compared. According to the clinical practice guidelines of the Orthopaedic Branch of the American Physical Therapy Association, the training program was divided into four parts. The first part is manual release of tense muscles, mainly including pectoralis major, pectoralis minor, levator scapulae, supraspinatus, subscapularis, and upper trapezius; the second part is to loosen the shoulder joints to increase the range of motion of the joints; the third part is to stretch the muscles, especially after the training, it needs to be stretched and relaxed in time. The last part is to strengthen the muscle strength of weak muscle groups, mainly including rhomboids, middle and lower trapezius, and infraspinatus. Factors that affect training load are shown in Figure 2.

### 3.6. Statistical Processing

#### 3.6.1. One-Way ANOVA

After the pairwise comparison test, be sure to carry out the post hoc test, also known as post hoc analysis, or called pairwise comparison analysis. Experimental data and measurement data are expressed as mean ± standard deviation (*x* ± *s*). SPSS13.0 software was used for statistical analysis. The comparison of EMG RMS values was carried out by the analysis of variance with two repeated measures factors (3 × 6), and the Geisser–Greenhouse correction coefficient was used to correct the degrees of freedom when the spherical test was not satisfied; additional subgroup test (post hoc) method was used to compare differences within groups. One-way ANOVA was used to compare the muscle strength parameters. If there was a significant difference, the SNK method was used for the comparison between any two groups when the homogeneity of variance was satisfied; Tamhane's T2 method was used to test when the requirement of homogeneity of variance was not met. The test standard was set at 0.05, the confidence interval was 95%, and *P* < 0.05 indicated a significant difference.

For the *i*th pair of matching points, the error term is defined as follows [12]:

(8) $$\begin{array}{c} e_{i}=p_{i}-\left(Rp+t\right),\\ \min J=\frac{1}{2}{\sum_{i=1}^{n}\left\|p_{i}-\left(Rp+t\right)\right\|}^{2}. \end{array}$$

For two sets of matching points, we define the centroid point as follows [13]:

(9) $$\begin{array}{c} p=\frac{1}{n}\sum \left(p_{i}\right),\\ p_{m}=\frac{1}{n}{\sum \left(p_{i}\right)}_{m}. \end{array}$$

So, the error function can be simplified to [14]

(10) $$\begin{array}{c} \min J=\frac{1}{2}\sum \left({\left\|p_{i}-p-R\left(P_{i}^{\prime }-p^{\prime }\right)\right\|}^{2}+{\left\|p_{i}-R\left(p-P_{i}^{\prime }-p^{\prime }\right)\right\|}^{2}\right). \end{array}$$

*q*_*i*_, *q*_*i*_′ are the decentroid coordinates of the two sets of points [15].

Hence [16], the equation is as follows:

(11) $$\begin{array}{c} \frac{1}{2}{\sum \left\|p_{i}-p-R\left(p-p^{\prime }\right)\right\|}^{2}=\frac{1}{2}{\sum \left\|p_{i}-p\right\|}^{2}. \end{array}$$

We define the matrix as follows [17]:

(12) $$\begin{array}{c} W=\sum q_{i}q_{i}^{T}. \end{array}$$

Available equation is as follows:

(13) $$\begin{array}{c} W=U\sum V^{T},\\ R=UV^{T}. \end{array}$$

## 4. Characteristics of Shoulder Joint Dysfunction in Volleyball Players and the Effect of Rehabilitation Training

### 4.1. Comparison Results between Groups

It can be seen from Table 1 that there was no difference in the SPADI (Shoulder Pain and Disability Index) scores of the athletes in the rehabilitation group and the rehabilitation control group before the intervention; there was no difference in the scores of athletes between the pre-rehabilitation and pre-rehabilitation control groups; the scores between the rehabilitation group and the pre-rehabilitation group were significantly different, *P* < 0.05. The SPADI score results after the end of the first week showed that the score of the rehabilitation group was lower than that of the rehabilitation control group, but there was no significant difference between the two groups. From the end of the second week to the end of the fourth week, the score of the rehabilitation group was significantly lower than that of the rehabilitation control group, *P* < 0.05; there was still no significant difference between the pre-rehabilitation group and the pre-rehabilitation control group. After the fourth week, the score gap between the rehabilitation group and the pre-rehabilitation control group was narrowed, and the score of the pre-rehabilitation control group increased, and there was no difference between the pre-rehabilitation group and the pre-rehabilitation group. The SPADI comparison results are given in Table 1.

### 4.2. Intragroup Comparison Results

With the progress of the intervention training, the scores of the rehabilitation group decreased continuously, and the scores from the end of the second week to the end of the fourth week were significantly different from those before the intervention, *P* < 0.05; the scores of the rehabilitation control group were also decreased, but there was no significant difference; although the pre-rehabilitation control group had no significant change before and after the intervention, there was an increasing trend. Changes in SPADI scores are shown in Figure 3.

### 4.3. Comparison Results between Groups

When the angular velocity was 60°/s, the peak flexor torque of the normal SPADI score group before intervention was greater than that of the abnormal score group. After the intervention, the difference in peak flexor torque between the rehabilitation group and the pre-rehabilitation group showed a decreasing trend, and the peak torque in the rehabilitation group was higher than that in the pre-rehabilitation control group. Before intervention, the peak extensor torque of the normal SPADI score group was greater than that of the abnormal group; after the intervention, the difference between the peak extensor torque of the rehabilitation group and the normal score group decreased, but it still did not reach the peak extensor torque level of the normal score group. When the angular velocity was 180°/s, the peak flexor torque of the normal SPADI score group before the intervention was greater than that of the abnormal score group. After the intervention, the difference between the peak flexor torque of the rehabilitation group and the normal score group decreased; the gap between the peak flexor torque of the rehabilitation control group and the normal score group has an increasing trend; the gap between the rehabilitation group and the rehabilitation control group, and the pre-rehabilitation and the pre-rehabilitation control group has an increasing trend. Before intervention, the peak extensor torque of the normal score group was greater than that of the abnormal group. After the intervention, the difference between the peak extensor torque of the rehabilitation group and the normal score group had a decreasing trend; the difference between the rehabilitation group and the rehabilitation control group, and the pre-rehabilitation and the pre-rehabilitation control group had an increasing trend. Isokinetic concentric flexion and extensor strength tests are shown in Figure 4.

### 4.4. Intragroup Comparison Results

It can be seen from the table that after the intervention in the rehabilitation group, the peak torque of the internal and external rotators has a tendency to increase. And with the increase of angular velocity, the peak torque decreases. After technical training and normal physical training, the peak torque of internal and external rotators in the rehabilitation control group decreased. After the intervention in the pre-rehabilitation group, the peak torque of the internal and external rotators showed an increasing trend. In the pre-rehabilitation control group, both internal and external rotators tended to increase after the intervention. Isokinetic concentric external rotation and internal rotation muscle strength test data are shown in Figure 5.

### 4.5. Intragroup Comparison Results

It can be seen that in the rehabilitation group, after the intervention, the peak torque of the abductor and adductors has an increasing trend, and with the increase of angular velocity, the peak torque decreases. In the rehabilitation control group, the peak torque of abductor and adductors decreased after technical training and normal physical training. In the pre-rehabilitation group, the peak torque of the abductor and adductors all tended to increase after the intervention. Changes in peak abductor and adductor muscle torque are shown in Figure 6.

Table 2 provides the root-mean-square amplitude values (microvolts) of the latissimus dorsi, biceps, triceps, and serratus anterior in the dysfunction group and the normal group before training, respectively. The root-mean-square amplitude value is an effective value reflecting muscle discharge. Its size is directly related to the change of the amplitude of the EMG signal and is closely related to the force generated during the air spiking of the target muscle. The RMS results under the serratus anterior and trapezius in the dysfunction group were significantly different from those in the normal group, and the dysfunction group was lower than the normal group; the RMS results in the trapezius muscle of the dysfunction group were significantly different from those of the normal function group, and the dysfunction group was lower than the normal function group. The RMS of the target muscle in the spiking action before training is given in Table 2.

The RMS results under the serratus anterior and trapezius were significantly improved in the functional disability group after rehabilitation training; the RMS results of the trapezius muscle were significantly improved compared with those before rehabilitation, and the RMS results of the other muscles had no significant difference but increased. The RMS (microvolts) of the target muscles in the spiking action of the dysfunction group before and after training is given in Table 3.

The degree of muscle activation under the serratus anterior and trapezius in the dysfunction group was significantly different from that in the normal function group, and the dysfunction group was lower than the normal function group; the degree of muscle activation in the trapezius muscle of the dysfunction group was significantly different from that of the normal function group, and the dysfunction group was lower than the normal function group; there was no significant difference in the degree of activation of other muscles, but the dysfunction group was lower than the normal function group. The muscle activation degrees (*M* ± SD) of the target muscles in the spiking action before training are given in Table 4.

The activation degree of the serratus anterior and the trapezius muscle in the functional disability group was significantly improved after rehabilitation training; the activation degree of trapezius muscle was significantly improved compared with that before rehabilitation, and the activation degree of other muscles had no significant difference but increased. The muscle activation degrees (*M* ± SD) of the target muscles in the spiking action of the dysfunction group before and after training are given in Table 5.

Whether the selection of evaluation indicators is reasonable or not affects the value of the entire research results. To this end, the selected indicators were evaluated by experts by means of a questionnaire on the recognition of expert indicators. According to the form of Richter scale, experts' recognition of these indicators is divided into 5 grades: very recognized, recognized, basically recognized, generally recognized, and not recognized, and assigned 5 points, 4 points, 3 points, 2 points, and 1 point, respectively. The evaluation results are given in Table 6.

The data of students and experts are summarized and analyzed, as shown in Figure 7, and the ranking of risk sources of sports injury technical action risk sources in sports volleyball special teaching activities is obtained: smash comes first, second is blocking, third is padding, fourth is passing, fifth is serving, and sixth is moving. It can be clearly seen from the figure that the risk of spiking and blocking is much higher than that of other technical action risk sources. The difference in risk amount of padding and passing is small, and movement is the smallest risk source of technical action risk sources.

Summarizing the data analysis of athletes and experts, it is concluded that the ranking of the risk sources of the main risk sources of sports injury athletes in sports volleyball special teaching activities is shown in Figure 8. Inherent injuries are ranked first, skills are second, physical ability is third, mental ability is fourth, tactical ability is fifth, self-management is sixth, and mental state is seventh. It can be clearly seen that the risk of inherent injuries and skills is much higher than that of other students' main risk sources. Physical fitness and mental ability have little difference in risk amount, and mental state is the smallest risk source among students' main risk sources.

According to the survey, the majority of volleyball coaches who have not participated in the training and study in the past three years account for the majority, which shows that the continuing training of volleyball coaches needs to be strengthened, and the training related to sports injuries should be paid more attention.  Figure 9 shows the volleyball coaches from different schools who participated in the training in the past three years.

## 5. Discussion

Volleyball is one of China's dominant sports and has created a glorious history in the world of volleyball. Maintaining the dominant position and sustainable development of the Chinese women's volleyball team is the main task of the development of Chinese competitive volleyball. Risk factors for sports teams to manage risk are as follows: unscientific work and rest time for athletes, neglect of cultural and ideological education for athletes, unscientific training time for athletes, lack of due diligence by field managers, problems with field equipment, and unclear division of labor or poor coordination among sports team managers. From the above risk factors, it can be seen that the management risk of sports teams often does not directly cause sports injuries, but affects sports training, learning, and life from a macro perspective, and affects other aspects through implication, such as the unscientific training time, which may affect the physical fitness of athletes [18, 19]. In order to keep the Chinese women's volleyball team as a world-class strong team, the State Sports General Administration has always attached great importance to the echelon construction of the women's volleyball team. They have built a relatively complete national volleyball high-level reserve talent base, women's volleyball team (hereinafter referred to as sports school women's volleyball team), the national youth women's volleyball team, and the national adult women's volleyball team, three different levels of women's volleyball echelons.

From the perspective of the characteristics of volleyball, competitive volleyball, as a comprehensive competitive sport, requires athletes to have comprehensive sports qualities, such as reaction, speed, strength, endurance, flexibility, and coordination. With the gradual development of artificial intelligence technology, the rapid progress of technology has promoted the rapid development of artificial intelligence technology in the field of sports. In China, the application of artificial intelligence technology in hospitals is also becoming more and more popular. With the continuous improvement of intelligent technology and the continuous improvement of application technology, the level of intelligence in the sports system will be higher and higher [20]. How to make training more scientific and targeted, scientifically and effectively regulate training, enhance strengths and complement weaknesses, avoid the risk of sports injuries, and ensure the steady improvement of Chinese women's volleyball players' competitive ability at different levels is the constant theme of volleyball scientific research.

Intelligent machines can make real-time judgments through experience and then perform specified behaviors and realize functional value [21, 22]. The representative technology at this stage is the intelligent program system of “expert system,” which covers a large number of human experts' knowledge and experience. Artificial intelligence can respond to real-time functional requirements according to a large amount of data in memory, and then execute commands [23–26].

## 6. Conclusion

Artificial intelligence improves the professional level and competitive ability of competitive sports: with the continuous in-depth application of data-driven sports training and sports decision making in developed countries, it has become a hot spot in the development of modern competitive sports. The time risk is mainly reflected in the change of training time, which causes the rhythm of the human body to change, which in turn affects the incompatibility of various abilities of the student's body and causes sports injuries. Referee risk, social support, and event arrangement risk are all factors that indirectly affect the risk of sports injuries. This work studies and analyzes the causes of abnormal postures and injuries of volleyball students and further analyzes the relationship between the two. Starting from the relationship between injury and abnormal posture of volleyball students, some preventive and restorative methods are proposed, but this research still needs to be improved and perfected.

## Figures and Tables

**Figure 1:** System's pass classification.

**Figure 2:** Factors affecting training load.

**Figure 3:** SPADI score changes.

**Figure 4:** Isokinetic concentric flexion and extensor strength test.

**Figure 5:** Isokinetic concentric external rotation and internal rotation muscle strength test data.

**Figure 6:** Changes in peak abductor and adductor muscle torque.

**Figure 7:** Summary analysis of student and expert data.

**Figure 8:** Ranking of risk sources of main risk sources for sports injuries in sports volleyball special teaching activities.

**Figure 9:** Volleyball coaches from different schools participated in training in the past three years.

**Table 1:** SPADI comparison results.

Group	Pre-intervention score	End of first week	End of second week	End of third week	End of fourth week
Rehabilitation group	7.45 ± 3.50	5.91 ± 2.88	3.82 ± 2.52	3.18 ± 2.44	2.91 ± 2.34
Rehabilitation control group	7.30 ± 4.08	7.20 ± 3.58	7.10 ± 3.45	7.30 ± 3.40	7.50 ± 2.51
Pre-rehabilitation	0 ± 0	0 ± 0	0.25 ± 0.71	0 ± 0	0.13 ± 0.35
Pre-rehabilitation control group	0 ± 0	0.13 ± 0.35	0.5 ± 0.93	0.63 ± 0.92	0.75 ± 0.89

**Table 2:** RMS of target muscles during spiking before training.

Muscle	Normal function group	Dysfunction group (*n* = 10)
Latissimus dorsi	193.56 ± 163.38	186.42 ± 145.19
Biceps	280.50 ± 110.92	273.35 ± 135.24
Triceps	255.33 ± 166.17	247.20 ± 159.37
Serratus anterior	207.85 ± 122.81	126.04 ± 61.58

**Table 3:** RMS (microvolts) of target muscles in the spiking action of the dysfunction group before and after training.

Muscle	Functional disability group before training	After training in the functional disability group
Latissimus dorsi	186.42 ± 145.19	191.22 ± 125.07
Biceps	273.35 ± 135.24	279.48 ± 156.61
Triceps	247.20 ± 159.37	254.39 ± 129.24
Serratus anterior	126.04 ± 61.58	248.56 ± 141.89

**Table 4:** Muscle activation of target muscles in spike action before training (*M* ± SD).

Muscle	Normal function group	Dysfunction group
Latissimus dorsi	0.122337187	0.121023957
Biceps	0.116638811	0.081346871
Triceps	0.165755966	0.094038219
Serratus anterior	0.108221821	0.121676154

**Table 5:** Muscle activation degree of target muscles in the spiking action in the dysfunction group before and after training (*M* ± SD).

Muscle	Normal function group	Dysfunction group
Latissimus dorsi	0.776050077	0.814957533
Biceps	0.709070941	0.72359654
Triceps	0.808669198	0.827771966
Serratus anterior	0.637256148	0.753439008

**Table 6:** Evaluation results.

Risk assessment indicators	Very recognized (5 points)	0 approval (4 points)	Basic approval (3 points)	General recognition (2 points)	Disapproved (1 point)
Possibility	12	0	0	0	0
Seriousness	12	0	0	0	0
Controllability	9	3	0	0	0
Persistent	8	2	2	0	0
Implicated	8	1	3	0	0

## Data Availability

Data sharing is not applicable to this article as no new data were created or analyzed in this study.
